# Research on Knee Joint Load and Influencing Factors of Typical Tai Chi Movements

**DOI:** 10.1155/2022/6774980

**Published:** 2022-03-08

**Authors:** Cenyi Wang, Ganfeng Yang, Haoping Yang, Changde Chen, Henrui Zhang, Kailong Wang, Aming Lu

**Affiliations:** ^1^School of Physical Education and Sports Science, Soochow University, Suzhou, China; ^2^First School of Clinical Medicine, Guangxi University of Chinese Medicine, Nanning, China

## Abstract

**Background:**

Tai chi is recognized worldwide for its rehabilitation abilities and healthcare benefits. However, in recent years, some movements associated with tai chi have been shown to damage the lower limb joints. The purpose of this study was to investigate and compare the effects of different movements, postures, center of mass (COM) movements, and range of knee movement of tai chi exercises on knee joint load.

**Methods:**

Fourteen professional tai chi practitioners in two postures (high and low) were enrolled to perform the following four typical tai chi movements: wild horse's mane (WHM), repulse monkey (RM), wave-hand in cloud (WHIC), and grasp the bird's tail (GBT). Kinematic and kinetics data were synchronously collected using the Vicon infrared high-speed motion capture system and a three-dimensional (3D) force measurement platform. Variance analysis and partial correlation analysis were performed to investigate factors influencing peak knee joint moment and vertical ground reaction force (VGRF).

**Results:**

The results showed that the peak knee extension and abduction moment were larger in WHM and RM than those in WHIC and GBT (*p* < 0.05). WHM was associated with greater rotation moment than the other typical movements (*p* < 0.05). VGRF and joint moment among different poses were significantly different. Low-pose tai chi typical movements were associated with greater VGRF, knee joint extension and abduction, and rotation moments than high-pose movements (*p* < 0.05). The anteroposterior and mediolateral COM displacements were strongly and positively associated with VGRF (*p* < 0.001), while the mediolateral COM displacement was negatively associated with knee extension moment (*p* < 0.001). The knee internal-external rotation ROM and anteroposterior and mediolateral COM displacements were positively associated with knee abduction moment (*p* < 0.01).

**Conclusion:**

For long-term tai chi exercises, choosing a suitable posture based on an individual exercise level and reasonable control of knee ROM and COM displacement can reduce the risk of knee injury during exercise.

## 1. Introduction

Tai chi is a classic traditional Chinese exercise inherited from ancient China, more than 2000 years ago. It is a core representative of Chinese culture for its profound self-healing and self-cultivation effects. It is characterized by coordinated body posture and movements, deep rhythmic and slow breathing, and mental focus. Tai chi is not only associated with physical and mental fitness but has also shown promising benefits as part of rehabilitation programs and is gradually being recognized worldwide [1].

The unique coordinated movements of tai chi are associated with significant effects on improving strength and endurance of the skeletal muscle and ameliorating proprioception and neuromuscular control function in older adults [2–4]. Previous studies have found that implementation of the push hands and wild horse's mane techniques of tai chi could be an optimal strategy to improve balance and prevent falls [5–7]. Compared with high pose, low-pose tai chi can elicit greater energy consumption and muscle activity [8, 9], thus leading to better exercise efficiency. However, with the popularization of tai chi and improvements in exercise techniques, there is a growing number of tai chi practitioners reporting knee joint pains or injuries after practicing tai chi. Studies have shown that nearly 40% of practitioners that did not have knee joint pain before practicing tai chi could eventually develop knee pain after long-term practice [10]. Thus, not all tai chi movements can be associated with beneficial effects on the joints of the lower limbs. This could be associated with the large amplitudes of lower limb movements and the long duration of weight-bearing and knee bending efforts during practice. Thus, compared with walking, studies have shown that tai chi movements such as squatting, pushing down, and lunges force the knee joint to exert more load on the sagittal and frontal plane [11], leading to knee pain, especially in elderly people. However, to our knowledge, there are also many studies showings the benefits of tai chi in ameliorating knee pains, and currently, there is a lack of studies investigating the relationship between specific tai chi movements or postures and knee pain.

In this study, we aimed to investigate the impact of specific tai chi movements on the knee joint of professional tai chi practitioners. We hypothesized that different tai chi movements would yield different knee range of motion (ROM) and center of mass (COM) displacements due to varying load intensities on the knee joint. The four classical movements of the 24-form simplified tai chi routine, namely, wild horse's mane (WHM), repulse monkey (RM), wave-hand in cloud (WHIC), and grasp the bird's tail (GBT), were selected to represent the four typical tai chi gaits: forward step, backward step, sidestep, and middle standing, respectively [12]. Thus, by comparing the knee joint load characteristics of these four movements in the high and low pose, we explore their influence on the lower limb joints COM displacement and ROM to deepen our understanding of the biomechanics of tai chi and provide a more scientific basis to tai chi practitioners on the associated risk of knee injury.

## 2. Methods

### 2.1. Participants

Based on a sample size calculation of the G∗Power 3.1 software, a total of fourteen participants, eight males and six females (age: 20.9 ± 1.2 years, height: 1.72 ± 0.07 m, and body mass: 67.5 ± 10.7 kg), were recruited for this study. All participants were tai chi training athletes from the College of Physical Education of Soochow University, were proficient in the 24-form simplified tai chi movements, had more than three years of professional training, and had participated in domestic and international tai chi events or large-scale competitions. The participants were in good health, had no history of knee injury, and had no major musculoskeletal injury of the lower limbs in the past year prior to study enrollment. This study protocol was reviewed and approved by the Ethics Committee of Soochow University (202104A331).

### 2.2. Instruments

Three-dimensional (3D) high-speed motion capture systems composed of eight infrared cameras (100 Hz, Vicon Motion Analysis, UK) and equipped with 35 tracking reflective markers with a diameter of 14 mm for motion capture and collection were used for this study. The position of marker adhesion was made following the standard protocol of the Plug-in Gait marker set [13]. Two force platforms (90 cm × 60 cm × 10 cm, model 9287B, Kistler Instrument Corp., Switzerland) were selected for mechanical testing. The sampling frequency was set to 1000 Hz and was synchronized with the Vicon infrared high-speed motion capture system. The position of the force platforms covered the plantar force area of the four investigated typical tai chi movements. The BioVision multichannel motion bioelectric recording and analysis system (BioVision, Germany) was used to monitor the knee flexion angle in real time.

### 2.3. Experimental Protocol

After the participants entered the examination room, the researchers first explained the whole process of the test to them and performed basic measurement, including recording of each participant's height, weight, and lower limb length. To reduce experimental error, the entire procedure was guaranteed to be completed by the same researcher. Before formally starting the experiment, each participant was given 5-10 min to practice the 24-form simplified tai chi as a warm-up routine and to familiarize with the experimental environment (Figure 1).

At the beginning of the experiment, the participants performed the four tai chi movements in different poses. The maximum knee flexion angle was assessed in real time using the BioVision multichannel motion bioelectric recording and analysis system, which was placed on the outside of the left knee joint to determine the tai chi pose. The low pose was defined as an angle of 60° ± 5° (Figure 2(a)), while the high pose was defined as a maximum knee flexion angle of 30° ± 5° of the supporting leg (Figure 2(b)) [14]. The four investigated tai chi movements included the forward step, backward step, sidestep, and middle standing, which are the most typical gait movements in tai chi [12]. The participants were given a 2-4 min resting time between each movement to avoid fatigue. The tai chi exercises were controlled by a metronome and performed at a speed of 30 bpm. The participants were instructed to step onto the force platform with only one foot at a time. Meanwhile, to ensure the fluency of the movement, the participants were required to start the exercise from the previous movement and stop at the next movement to simultaneously collect kinematic and kinetic outcomes. The data of each typical tai chi movement and two postures were recorded and repeated three times for analysis.

### 2.4. Data Processing and Analysis

The Plug-in Gait full-body model (Oxford Metrics, UK) was implemented to calculate the 3D kinematics and kinetics data using Vicon Nexus (Oxford Metrics, UK) and Visual 3D (C-Motion, USA) software. Considering that the four investigated typical tai chi movements were symmetrical, the biomechanical characteristics of the left lower limb were selected to replace the entire movement. The main kinematic parameters selected were the COM displacement on three coordinate axes, the maximum knee flexion angle, and the knee ROM in three planes. The knee joint angle in the normal upright state of the human body was considered to be at 0 degrees. The peak joint moments in three directions of the left knee joint and the peak vertical ground reaction force (VGRF) during the support phase were selected as the kinetics parameters. A complete support phase was defined as the time when the left heel (left toe) contacted the ground and ended when the left toe (left heel) was off the ground. The support phase was 100% standardized. The definition of the heel (toe) contacting or leaving the ground was measured using the Vicon system to obtain the time when the left foot contacted and left the force platform and was supplemented by a visual inspection of the virtual heel and toe kinematic positions. After three repetitions, each participant's joint moment and VGRF in all directions were averaged and standardized according to their corresponding body weight in units of N·m/kg and BW, respectively. The COM displacement in the three directions of the sagittal axis, frontal axis, and vertical axis, measured in mm, was obtained by subtracting the minimum value from the maximum value of the COM.

### 2.5. Statistical Analysis

Descriptive statistics were performed using the SPSS 20.0 statistical software (SPSS Science, Chicago, USA), and the Shapiro-Wilk test was used to verify the normal distribution of continuous variable. The normality of the distribution of continuous variables was examined using the Shapiro-Wilk test. All data were described in the form of the mean ± standard deviation (M ± SD). A 4 × 2 (movement × pose) repeated measures analysis of variance (ANOVA) was used to examine the effect of each categorical variable on the selected dependent variable: joint moment and VGRF. Post hoc comparisons using paired sample *t*-tests were performed with Bonferroni adjustments to determine the differences between each movement. Bivariate correlation analysis and partial correlation analysis were used to investigate the correlation between each continuous variable and the selected dependent variable. The significance level was set at *α* = 0.05.

## 3. Results

### 3.1. The Effect of Pose and Movement on Knee Joint Load

#### 3.1.1. The Effect of Pose and Movement on Peak VGRF

The peak VGRF value of the four movements in different poses was statistically significant (Table 1). The peak VGRF value of each movement in the low pose was greater than that in the high pose. Compared with the other three movements of tai chi, GBT had a significantly smaller peak VGRF value in both poses.

#### 3.1.2. The Effect of Pose and Movement on Peak Knee Moment

The peak knee moment of each classical tai chi movement in different poses was statistically significant (Table 1). The knee extension moments of each movement in the low pose were significantly greater than the knee extension moment in the high pose. The knee extension moment of the WHIC movement in the high and low pose was significantly smaller than the other three movements. In regard to knee abduction moment, the values of all three movements in low pose were greater than those in high pose, except for WHM. Moreover, the knee abduction moments of WHIC and GBT in the high and low pose were significantly smaller than those of WHM and RM. In regard to knee rotation moment, except for RM, the values of the other three movements in low pose were greater than those in high pose. The knee external rotation moments of WHM and GBT were greater in low pose than in high pose, and the knee internal rotation moment of RM in low pose was smaller than those of WHM and GBT.

Regarding the dynamic trend characteristics of knee joint moments during the stance phase, on the sagittal plane, the time taken for the WHIC and GBT movements to reach their peak extension moment was significantly shorter than those of WHM and RM (Figure 3). On the frontal plane, the peak knee adduction and abduction moments of RM and WHIC occurred in the middle of the support phase, and compared with the other two movements, the peak support time of WHM and GBT was shorter (Figure 4). On the transverse plane, the peak rotation moments of WHM and GBT both occurred in the middle of the support phase, and the support time of GBT to reach the maximum knee external rotation moment was significantly shorter than the other three movements (Figure 5).

### 3.2. The Effect of Knee Joint ROM and COM Displacement on Knee Joint Load

#### 3.2.1. Correlation Analysis of Knee Joint ROM and COM Displacement

Table 2 shows the results of bivariate correlation analysis between the knee joint ROM and the displacement of the COM.

#### 3.2.2. Partial Correlation Analysis of Knee Joint ROM and COM Displacement to the Knee Joint Load

The partial correlation analysis results of knee joint load, based on variance analysis and bivariate correlation analysis [15], are presented in Table 3. The results show that the knee ROM and COM displacements of knee joint load were correlated with peak VGRF and knee moment. COM displacement in the anteroposterior and mediolateral directions was strongly and positively correlated with peak VGRF (*r* = 0.85; *r* = 0.88), while the mediolateral COM displacement was negatively correlated with extension moment (*r* = −0.57). The internal and external rotation motion of the knee joint and mediolateral COM displacement demonstrated a weak positive correlation with knee abduction moment. We also observed a strong positive correlation between the anteroposterior COM displacement and knee abduction moment (*r* = 0.77) and a negative correlation between the anteroposterior COM displacement and the knee external rotation moment (*r* = −0.60).

## 4. Discussion

### 4.1. Analysis of the Effect of Tai Chi Movements on Knee Joint Load

The results illustrate that different typical tai chi movements had significantly different effects on knee joint load. Previous studies have shown that compared with walking, tai chi was associated with a wider range of joint motion and a smaller peak VGRF value. Therefore, compared with walking, tai chi exercises could increase lower limb muscle strength without increasing lower limb joint load [12, 16, 17]. However, in this study, we noted significant differences in VGRF among the tai chi movements. Further, studies have confirmed that the position and speed of foot landing could affect GRF, and thus, the slow and gentle movements of tai chi would produce a lower VGRF ([6]), of which RM movements using the forefoot landing and WHIC using the outside foot landing would have a lower VGRF than WHM with the heel landing. In this study, we observed that the VGRF of RM and WHIC movements were between 1.03-1.04 N/BW and 1.03-1.05 N/BW, respectively, while the VGRF of WHM was between 1.05-1.07 N/BW, which were consistent with the findings of the previous studies [16, 18]. Thus, higher VGRF significantly increases the load on lower limb joints and induces knee pain [19], and excessive knee joint moments increase overall load on knee joint and directly damage its structure [20].

The peak knee extension and abduction moment are related to an increased load in the medial compartment of the knee joint and defect of the medial tibial cartilage, and excessive rotation moment of the knee joint could easily cause lateral displacement of the patella and lead to patellar ligament injury [8, 21, 22]. According to the results of this study, the peak knee extension moments of WHM, RM, and GBT movements were larger than those of WHIC, and the peak abduction moments of WHM and RM movements were more significant than those of WHIC and GBT. Further, we also observed a dynamic trend of knee joint moment during one support phase of the four tai chi movements. A high load rate may cause rapid deformation of joint tissues such as the articular cartilage, which may easily lead to premature aging or damage of the joint soft tissues, while a low load rate could allow the surrounding skeletal muscles and ligaments to buffer the peak force exerted on the joint to stabilize it [23]. Tai chi movements seem to be consistent with the viscous characteristics of human biological soft tissues. However, based on the observations from Table 1 and Figure 3, the peak knee flexion and extension moments in WHM, RM, and GBT movements were 400% greater than those of WHIC. Studies have found that the relatively high knee joint observed during tai chi lunge and pushdowns was due to a group of knee extensor muscles that play a vital role in maintaining a more flexed position of the knee joint [11], Thus, since WHM, RM, and GBT movements consist of lunges, especially the GBT movement, which consists of multiple lunges and pushdowns, this explains the larger values observed in contrast to WHIC. Hence, tai chi practitioners with weak muscle strength of the lower limb, especially the elderly, should pay attention to slow down the speed of reaching several peak moments when practicing such movements to prevent movement deformation, thus reducing the risk of knee joint injury [24].

### 4.2. Analysis of the Effect of Tai Chi Pose on Knee Joint Load

We also examined the influence of posture height of typical tai chi movements on the load of knee joint. Our results showed that for the same movement, the low pose had greater peak VGRF and knee extension, abduction, and rotation moment than the high pose. Low-pose tai chi is usually widely used by professional martial arts athletes or people with higher athletic abilities, while the high pose is more commonly used by the general population [9, 25]. Further, we found that in the low pose, the knee extension moments of the four typical tai chi movements were significantly greater than those of the corresponding movements in the high pose (Table 1). Considering that this might be related to the greater VGRF of each movement in the lower pose than that of high pose, this suggests that the extension moment and VGRF of the four movements could be dependent on the pose performed. According to the principle of the screw-home mechanism and related studies, the contact area between the tibial plateau and the meniscus of the knee joint is in the front when flexing between angles of 0° and 60°. After 60°, a continuous increase in the flexion angle increases the range of rotation, and the contact area between the tibial plateau and meniscus gradually shifts from the front to the rear, leading to a continuous increase in the contact stress between the tibial-femoral joint [26, 27]. The above conclusion corroborates with our findings which showed that the four movements of low-pose tai chi had larger peak VGRF values than those of high pose and further explain the impact of low-pose tai chi on the risk of injury to the medial knee joint meniscus. In addition, we also observed that the high pose had lower knee abduction moment than the low pose (Table 1). Although some researchers have pointed out that tai chi exercises have a lower knee abduction moment than normal walking [28], the results of this study showed that the choice of tai chi posture had a significant impact on the knee joint load, which may cause a great difference in the exercise effect compared with the expected one.

### 4.3. Analysis of the Effect of Knee ROM and COM Displacement on Knee Joint Load

In tai chi exercises, the maximum flexion angle of the knee joint is strongly associated with the height of the posture employed. Partial correlation analysis of this study showed that larger maximum knee flexion angle was associated with a larger peak knee extension moment, which also confirms that a lower pose was associated with a larger knee extension moment than a higher pose. Moreover, several studies have indicated that the depth of knee flexion was highly correlated with knee extension moment, and in order to complete movement in a lower posture, the knee extensor muscles should contract more to increase torque output [29, 30]. Consequently, for people with knee injuries or weak lower limb muscle strength, such as the elderly, movements requiring excessive knee flexion angle should not be recommended for daily tai chi practice. Additionally, the results of this study also showed that the peak knee abduction moment was related to the internal and external rotation of the knee joint, and the abduction moment of the knee joint increased with an increase in the knee internal and external rotation ROM. Hence, it is suggested to avoid excessive knee internal and external rotation activities to reduce knee injury or pain when practicing low-pose tai chi.

In this study, partial correlation analysis was performed to investigate the association between COM displacement and knee joint load in each direction. The results revealed that the anteroposterior COM displacement was highly correlated with the peak knee abduction moment and VGRF and correlated with the knee flexion and external rotation moment. Among the four typical movements selected in this study, WHM and RM movements represented the forward and backward displacements. Tai chi movements require the body to shift its center of gravity downward. While performing a downward movement and maintaining a low body center of gravity, to smoothly and stably transfer the center of gravity in a front-to-back direction, greater abduction, adduction, and rotation of knee joint are achieved by highly coordinated control of the muscles around the knee joint [31]. On the other hand, results of the partial correlation analysis showed that the mediolateral COM displacement was highly correlated with peak VGRF and correlated with the peak abduction, internal rotation, and extension moment of the knee. In this regard, WHIC, as a sidestep movement, is performed by moving the body in a relatively small distance via forward and backward movements and transfer of the center of gravity in the mediolateral directions. As this sidestep movement requires the hip and knee joints to perform sufficient abduction, adduction, and rotation during the tai chi movements, this may be the reason why the peak knee abduction and internal rotation moment increases with increase in mediolateral COM displacement while the knee extension moment decreases.

In contrast to previous studies, which tended to choose elderly or nonprofessional persons with long-term tai chi experiences to conduct tai chi biomechanics research [17, 28, 32, 33], in this study, we selected professional tai chi practitioners to allow uniform assessment of the selected four typical tai chi movements in different poses. We observed that even with such relatively uniform tai chi movements, different movements and poses and different knee ROM and COM displacements significantly impacted knee joint load. Despite the important findings shown in this study, there were some limitations. First, the gender of the subjects was not separately analyzed, and it is unclear whether gender difference could have affected our observations. Second, this study required the participants to make contact with the force platform with only one foot in each test. Although we instructed the participants to practice such movements several times to familiarize themselves with experimental settings, it cannot be guaranteed that such nondaily settings and environments could affect the stability of the movements. Furthermore, the results of knee rotation angle on the transverse plane in this study could have been overestimated, due to the presence of more rotation components in tai chi movements, and the abduction moment adopted in this study might not directly reflect the actual load of on knee medial compartment. Thus, future studies could consider incorporating musculoskeletal modeling approaches to evaluate the real impact of tai chi movements on knee joints in different poses.

## 5. Conclusion

In this study, significant differences between the knee joint loads of relatively standardized typical tai chi movements were observed and were significantly correlated with knee ROM and COM displacement. Therefore, it is recommended that tai chi practitioners should choose an appropriate posture based on their physical ability and health condition to reasonably control the range of knee joint motion and COM displacement during tai chi to reduce the impact of knee joint load, increase the benefits from these movements, and reduce the risk of knee joint injury.

## Figures and Tables

**Figure 1:** Lateral view of forward step: wild horse's mane (a); backward step: repulse monkey (b); sidestep: wave-hand in cloud (c); middle standing: grasp the bird's tail (d). The arrow indicates the direction of movement.

**Figure 2:** Peak knee flexion angle (left knee): (a) *α* = 60 ± 5° for low pose. (b) *α* = 30 ± 5° for high pose.

**Figure 3:** Joint moment at knee in sagittal plane in high (black) and low (gray) pose for wild horse's mane (WHM), repulse monkey (RM), wave-hand in cloud (WHIC), and grasp the bird's tail (GBT) during one support phase (*N* = 14). ^∗^*p* < 0.05.

**Figure 4:** Joint moment at knee in frontal plane in high (black) and low (gray) pose for wild horse's mane (WHM), repulse monkey (RM), wave-hand in cloud (WHIC), and grasp the bird's tail (GBT) during one support phase (*N* = 14). ^∗^*p* < 0.05.

**Figure 5:** Joint moment at knee in transverse plane in high (black) and low (gray) pose for wild horse's mane (WHM), repulse monkey (RM), wave-hand in cloud (WHIC), and grasp the bird's tail (GBT) during one support phase (*N* = 14). ^∗^*p* < 0.05.

**Table 1:** Mean and standard deviation of the peak vertical ground reaction force (VGRF) and joint moment of the left knee joint in the tai chi typical movements under different poses (VGRF unit: N/BW; moment unit: N·m/kg).

Variables	Pose	Pose effect	Wild horse's mane	Repulse monkey	Wave-hand in cloud	Grasp the bird's tail	Movement effect	Interaction
VGRF	High	*F*(1, 13) = 64.974, *p* < 0.001	1.05 ± 0.03^d^	1.03 ± 0.01^d^	1.04 ± 0.02^d^	0.70 ± 0.04^abc^	*F*(3, 39) = 605.948, *p* < 0.001	*F*(3, 39) = 5.124, *p* = 0.004
	Low		1.07 ± 0.02^∗^^bd^	1.04 ± 0.02^∗^^ad^	1.05 ± 0.02^∗^^d^	0.74 ± 0.04^∗^^abc^		
Flexion	High	*F*(1, 13) = 14.983, *p* = 0.002	0.32 ± 0.20^d^	0.28 ± 0.05^d^	0.21 ± 0.20	0.14 ± 0.05^ab^	*F*(1.944,25.268) = 3.841, *p* = 0.017	*F*(3, 39) = 1.337, *p* = 0.276
	Low		0.40 ± 0.16^d^	0.33 ± 0.14	0.28 ± 0.25^∗^	0.27 ± 0.08^∗^^a^		
Extension	High	*F*(1, 13) = 121.632, *p* < 0.001	0.51 ± 0.28^c^	0.52 ± 0.11^c^	0.11 ± 0.13^abd^	0.501 ± 0.18^c^	*F*(3, 39) = 19.259, *p* < 0.001	*F*(3, 39) = 11.122, *p* < 0.001
	Low		0.75 ± 0.30^∗^^c^	0.76 ± 0.24^∗^^c^	0.14 ± 0.17^∗^^abd^	0.83 ± 0.22^∗^^c^		
Abduction	High	*F*(1, 13) = 17.736, *p* = 0.001	0.94 ± 0.23^cd^	0.90 ± 0.18^cd^	0.23 ± 0.21^ab^	0.29 ± 0.08^ab^	*F*(3, 39) = 58.657, *p* < 0.001	*F*(1.554,20.204) = 0.593, *p* = 0.623
	Low		1.11 ± 0.39^cd^	1.02 ± 0.19^∗^^cd^	0.35 ± 0.28^∗^^ab^	0.36 ± 0.11^∗^^ab^		
Adduction	High	*F*(1, 13) = 82.841, *p* < 0.001	0.21 ± 0.08^b^	0.10 ± 0.06^a^	0.11 ± 0.12	0.15 ± 0.09	*F*(3, 39) = 9.327, *p* < 0.001	*F*(3, 39) = 7.796, *p* < 0.001
	Low		0.36 ± 0.10^∗^^bc^	0.18 ± 0.10^∗^^ad^	0.17 ± 0.17^∗^^ad^	0.35 ± 0.12^∗^^bc^		
Internal rotation	High	*F*(1, 13) = 44.170, *p* < 0.001	0.10 ± 0.06	0.05 ± 0.03	0.05 ± 0.04	0.05 ± 0.04	*F*(1.212,15.755) = 3.599, *p* = 0.070	*F*(3, 39) = 3.370, *p* = 0.028
	Low		0.21 ± 0.10^∗^^b^	0.07 ± 0.04^ad^	0.14 ± 0.10^∗^	0.16 ± 0.06^∗^^b^		
External rotation	High	*F*(1, 13) = 40.335, *p* < 0.001	0.30 ± 0.11^cd^	0.33 ± 0.09^cd^	0.13 ± 0.15^abd^	0.17 ± 0.02^abc^	*F*(3, 39) = 5.115, *p* = 0.004	*F*(3, 39) = 5.115, *p* = 0.004
	Low		0.49 ± 0.14^∗^^cd^	0.44 ± 0.13^cd^	0.22 ± 0.25^abd^	0.24 ± 0.05^∗^^abc^		

^a^Significant difference from wild horse's mane in the same pose, *p* < 0.05. ^b^Significant difference from repulse monkey in the same pose, *p* < 0.05. ^c^Significant difference from wave-hand in cloud in the same pose, *p* < 0.05. ^d^Significant difference from grasp the bird's tail in the same pose, *p* < 0.05. ^∗^Significant differences between the low pose and high pose in same movement, *p* < 0.05.

**Table 2:** Correlation analysis of knee joint range of motion (ROM) and center of mass (COM) displacement on knee joint load.

Continuous variable	Vertical GRF		Flexion moment		Extension moment		Abduction moment		Adduction moment		Int. rotation moment		Ext. rotation moment	
	*r*	*p*	*r*	*p*	*r*	*p*	*r*	*p*	*r*	*p*	*r*	*p*	*r*	*p*
Maximum knee flexion angle	0.10	n.s.	**-0.24**	0.012	**0.31**	0.001	0.13	n.s.	**-0.43**	<0.001	**0.31**	0.001	**-0.30**	0.001
Flexion and extension ROM	0.07	n.s.	**-0.25**	0.007	**0.39**	<0.001	**0.29**	0.002	**-0.47**	<0.001	**0.27**	0.004	**-0.39**	<0.001
Abduction and adduction ROM	0.13	n.s.	-0.01	n.s.	0.08	n.s.	0.10	n.s.	-0.08	n.s.	0.04	n.s.	-0.10	n.s.
Int. and ext. rotation ROM	**0.20**	0.035	**-0.27**	0.004	0.09	n.s.	**0.35**	<0.001	**-0.28**	0.003	**0.26**	0.007	**-0.34**	<0.001
COM: *X* (mm)	**0.33**	<0.001	**-0.32**	0.001	**0.55**	<0.001	**0.79**	<0.001	**-0.23**	0.016	-0.13	n.s.	**-0.71**	<0.001
COM: *Y* (mm)	**0.50**	<0.001	-0.06	n.s.	**-0.61**	<0.001	**-0.24**	0.011	0.08	n.s.	**0.37**	<0.001	**0.33**	<0.001
COM: *Z* (mm)	-0.13	n.s.	**-0.26**	0.006	**0.30**	0.001	0.17	n.s.	**-0.41**	<0.001	**0.31**	0.001	**-0.29**	0.002

Int.: internal; Ext.: external. Bold values indicate significant differences, *p* < 0.05. n.s. indicates nonsignificant differences.

**Table 3:** Partial correlation analysis of knee joint range of motion (ROM) and center of mass (COM) displacement on knee joint load.

Continuous variable	Vertical GRF		Flexion moment		Extension moment		Abduction moment		Adduction moment		Int. rotation moment		Ext. rotation moment	
	*r*	*p*	*r*	*p*	*r*	*p*	*r*	*p*	*r*	*p*	*r*	*p*	*r*	*p*
Maximum knee flexion angle	0.10	n.s.	-0.13	n.s.	**0.25**	0.010	-0.04	n.s.	-0.14	n.s.	0.08	n.s.	**-0.20**	0.038
Flexion and extension ROM	-0.09	n.s.	0.11	n.s.	0.02	n.s.	0.01	n.s.	-0.09	n.s.	0.01	n.s.	0.08	n.s.
Abduction and adduction ROM	-0.06	n.s.	0.14	n.s.	0.12	n.s.	-0.03	n.s.	-0.01	n.s.	-0.08	n.s.	0.03	n.s.
Int. and ext. rotation ROM	0.02	n.s.	-0.12	n.s.	-0.04	n.s.	**0.32**	0.001	-0.10	n.s.	0.10	n.s.	**-0.23**	0.018
COM: *X* (mm)	**0.85**	<0.001	**-0.36**	<0.001	**0.22**	0.021	**0.77**	<0.001	-0.04	n.s.	-0.04	n.s.	**-0.60**	<0.001
COM: *Y* (mm)	**0.88**	<0.001	**-0.23**	0.020	**-0.57**	<0.001	**0.27**	0.005	0.09	n.s.	**0.28**	0.003	0.06	n.s.
COM: *Z* (mm)	-0.09	n.s.	-0.13	n.s.	0.12	n.s.	-0.12	n.s.	-0.15	n.s.	0.18	n.s.	-0.03	n.s.

Int.: internal; Ext.: external. Bold values indicate significant differences, *p* < 0.05. n.s. indicates nonsignificant differences.

## Data Availability

The data used to support the findings of this study are included within the article.

## References

[1] Hong Y., Li J. X., Robinson P. D. (2000). Balance control, flexibility, and cardiorespiratory fitness among older tai chi practitioners. *British Journal of Sports Medicine*.

[2] Cheng L., Chang S., Li J., Hong Y. (2017). Effects of different periods of tai chi exercise on the kinesthesia of the lower limb joints of elderly women. *Research in Sports Medicine (Print)*.

[3] McGibbon C. A., Krebs D. E., Parker S. W., Scarborough D. M., Wayne P. M., Wolf S. L. (2005). Tai chi and vestibular rehabilitation improve vestibulopathic gait via different neuromuscular mechanisms: preliminary report. *BMC Neurology*.

[4] Penn I. W., Sung W. H., Lin C. H., Chuang E., Chuang T. Y., Lin P. H. (2019). Effects of individualized tai-chi on balance and lower-limb strength in older adults. *BMC Geriatrics*.

[5] Chen H. C., Cheng K. Y., Liu Y. J., Chiu H. T., Cheng K. Y. (2010). The defence technique in tai chi push hands: a case study. *Journal of Sports Sciences*.

[6] Law N. Y., Li J. X. (2014). The temporospatial and kinematic characteristics of typical tai chi movements: repulse monkey and wave-hand in cloud. *Research in Sports Medicine (Print)*.

[7] Yang F., Liu W. (2021). Individual analysis of dynamic stability for twenty-four tai chi forms among persons with knee osteoarthritis: a pilot study. *Gait & Posture*.

[8] Xiao Y. (2020). *The Effects of Muscle Activity and Joint Load in Patients with Knee Osteoarthritis on Different Positions of Tai Chi Movement: Wave-Hand in Cloud*.

[9] Yang H., Yu D., Zhao Y. (2011). Gaseous metabolism and expenditure of energy in the process of TaiJiQuan’s Yemafenzong, Daojuangong and Yunshou movements exercise of the elderly men. *Chinese Journal of Sports Medicine*.

[10] Zhu D., Li L., Qiu P., Wang S., Xie Y., Chen X. (2011). Investigation and analysis of knee joint pain in Taijiquan practitioners in Shanghai. *Chinese Journal of Sports Medicine*.

[11] Wen C., Zhang S., Cao X., Zhang Y., Crouter S. E., Wozencroft A. J. (2015). Knee biomechanics of selected knee unfriendly movement elements in 42-form tai ji. *Medicine & Science in Sports & Exercise*.

[12] Mao D. W., Hong Y., Li J. X. (2006). Characteristics of foot movement in tai chi exercise. *Physical Therapy*.

[13] Davis R. B., Unpuu S., Tyburski D., Gage J. R. (1991). A gait analysis data collection and reduction technique. *Human Movement Science*.

[14] Zhou L., Wang J., Wu F., Lin X. (2005). Determination and control of three postures of Taijiquan. *China Sport Science and Technology*.

[15] Zhao F., Liu T. (2016). Application of partial correlation analysis in the study of pulse pressure correlation factors. *Chinese Journal of Health Statistics*.

[16] Li J. X., Law N. Y. (2018). Kinetics of the lower limb during two typical tai chi movements in the elderly. *Research in Sports Medicine (Print)*.

[17] Wong S. H., Ji T., Hong Y., Fok S. L., Wang L. (2013). Foot forces induced through tai chi push-hand exercises. *Journal of Applied Biomechanics*.

[18] Wang H., Ji Z., Zhang Z., Pang B., Zhang C. (2019). Biomechanical characteristics of lower limbs in 24-form taichi movement. *Journal of Chengdu Sport University*.

[19] Radin E. L., Yang K. H., Riegger C., Kish V. L., O'Connor J. J. (1991). Relationship between lower limb dynamics and knee joint pain. *Journal of Orthopaedic Research : Official Publication of the Orthopaedic Research Society*.

[20] Tao P., Yu L. (2014). The comparison of knee joint kinematics, joint load and muscle activity characteristics for tai chi basic action “the wild horse’s mane on both side”. *China Sport Science*.

[21] Messier S. P., Beavers D. P., Mihalko S. L. (2020). The effects of intensive dietary weight loss and exercise on gait in overweight and obese adults with knee osteoarthritis. The Intensive Diet and Exercise for Arthritis (IDEA) trial. *Journal of Biomechanics*.

[22] Xu W., Li Y. (2008). On Yang Taijiquan performers’ outward shift of kneecaps and corresponding correctness. *Journal of Beijing Sport University*.

[23] Quinn T. M., Allen R. G., Schalet B. J., Perumbuli P., Hunziker E. B. (2001). Matrix and cell injury due to sub-impact loading of adult bovine articular cartilage explants: effects of strain rate and peak stress. *Journal of Orthopaedic Research : Official Publication of the Orthopaedic Research Society*.

[24] Zhu Y. (2002). The cause and prevention of knee joint injury in hexagram boxing exercises. *Journal of Sports Sciences*.

[25] Chen W., Zhao F. (1984). Changes of energy consumption and nail wrinkle microcirculation in Taijiquan practice. *Journal of Shanghai University of Sport*.

[26] Jeon J. W., Hong J. (2021). Comparison of screw-home mechanism in the unloaded living knee subjected to active and passive movements. *Journal of Back and Musculoskeletal Rehabilitation*.

[27] Zhang L. K., Wang X. M., Niu Y. Z., Liu H. X., Wang F. (2016). Relationship between patellar tracking and the “screw-home” mechanism of tibiofemoral joint. *Orthopaedic Surgery*.

[28] Liu W., Kovaleski J. E., Kepple T. M. (2016). DoesT'ai ChiGait reduce external knee adduction moment?. *Journal of Alternative and Complementary Medicine (New York, N.Y.)*.

[29] Creaby M. W., Hunt M. A., Hinman R. S., Bennell K. L. (2013). Sagittal plane joint loading is related to knee flexion in osteoarthritic gait. *Clinical Biomechanics (Bristol, Avon)*.

[30] Jenkyn T. R., Hunt M. A., Jones I. C., Giffin J. R., Birmingham T. B. (2008). Toe-out gait in patients with knee osteoarthritis partially transforms external knee adduction moment into flexion moment during early stance phase of gait: a tri-planar kinetic mechanism. *Journal of Biomechanics*.

[31] Gao Q. (2020). *Biomechanical analysis of typical movements of tai chi and its enlightenment in physical education*.

[32] Duan J., Wang K., Chang T., Wang L., Zhang S., Niu W. (2019). Tai chi is safe and effective for the hip joint: a biomechanical perspective. *Journal of Aging and Physical Activity*.

[33] Yang F., Liu W. (2020). Biomechanical mechanism of tai-chi gait for preventing falls: a pilot study. *Journal of Biomechanics*.

